# Addressing the Evidence Gap: Protocol for an Effectiveness Study of Circle of Security Parenting, an Attachment-Based Intervention

**DOI:** 10.3389/fgwh.2020.575752

**Published:** 2020-10-22

**Authors:** Anne-Marie Maxwell, Catherine McMahon, Anna Huber, Erinn Hawkins, Rebecca Elizabeth Reay

**Affiliations:** ^1^Department of Psychology, Centre for Emotional Health, Macquarie University, Sydney, NSW, Australia; ^2^School of Applied Psychology, Menzies Health Institute Queensland, Griffith University, Gold Coast, QLD, Australia; ^3^ANU Medical School, Academic Unit of Psychiatry and Addiction Medicine, Australian National University, Canberra, ACT, Australia

**Keywords:** Circle of Security Parenting (COS-P), parenting education, attachment-based intervention, caregiving representations, parent mentalization

## Abstract

**Background:** Parenting interventions informed by attachment theory are an increasingly popular choice for clinical services that work with parents of babies and young children. Circle of Security Parenting (COS-P) is one such intervention, which has had extraordinary uptake internationally. Evidence for COS-P is very limited, however; there are few published studies, most with very small samples, and findings are mixed. This paper describes a multi-site evaluation of COS-P, designed to help address this evidence gap.

**Methods/Design:** This is a non-randomized controlled effectiveness study of COS-P in four community child and family health settings. Participants are caregivers of children aged 6 years and under, who present to study sites with parenting challenges in the early parenting period. Participants are recruited through these sites, and allocated to either treatment or waitlist control condition based on their capacity to attend the next available COS-P group. Outcomes (changes in caregiving attitudes and capacities linked to child social and emotional development, and caregiver depression symptoms) are assessed at baseline and post-treatment/waitlist using self-report questionnaires (all participants), and a narrative interview and 5-min parent-child interaction (a sub-sample of participants). Additionally, potential moderators of the intervention (demographic, symptom severity) will be tested.

**Discussion:** This is one of the first controlled evaluations of COS-P, and the first in Australia where COS-P dissemination has been particularly widespread. Results from this study will provide valuable information about the effectiveness of COS-P for caregivers with early parenting challenges, and will increase understanding of what works for whom.

## Introduction

Attachment theory (1–3) has informed thinking and practice in infant mental health for decades (4). It is also increasingly influential within the broader field of early childhood service provision (5). Parenting interventions based on attachment theory seek to improve the quality of the parent-child relationship and thus to improve the child's developmental trajectory, particularly with respect to social-emotional development. One of the most widely disseminated attachment-based interventions is Circle of Security Parenting (COS-P) (6, 7), an 8-week program that aims to build parenting capacity in parents of children aged from approximately 6 months to 6 years (7). COS-P is based on a more intensive 20-week Circle of Security protocol (8, 9), that allows individualized therapeutic work utilizing video feedback. COS-P was developed to facilitate broader implementation and uses stock DVD footage in place of individualized video material to demonstrate important concepts relevant to supporting secure attachment relationships (10). The centerpiece of both versions is a simple graphic (Figure 1), which captures the core dynamic at the heart of attachment theory regarding the child's need for both connection and exploration, and the caregiving behaviors that support these needs (11–13). Also fundamental to both versions is the therapeutic relationship between facilitator and participants (14).

**Figure 1:** Circle of Security circle graphic. Copyright 2016 by Cooper, Hoffman, and Powell. Reproduced with permission.

COS-P is broadly disseminated in North America, Europe, and Asia, and has proved particularly popular in Australia, where more than 10,000 COS-P facilitators had been trained by late 2016 (14). This figure will now be substantially higher, with more than 10 official COS-P training courses held around the country each year, often training more than 200 individuals at a time. Several state government departments and large non-profit organizations have adopted COS-P and/or the overarching COS model to inform their work with families of young children. Surprisingly, however, evidence for COS has not kept pace with dissemination (5), with remarkably few evaluation studies published to date for either version, precluding their endorsement as evidence-based programs by bodies like the influential California Evidence-Based Clearinghouse for Child Welfare (15).

Two studies of the intensive COS-I intervention with pre-post-designs have shown improvement in indices of child attachment in U.S. (13) and Australian (16) samples. The second of these studies also showed an increase in caregiver reflective functioning and caregivers' positive caregiving representations (16), improvements in child behavior problems and child social-emotional protective factors (17), and reductions in parenting stress and parent mental health symptoms (18). While these results are encouraging and in line with theory, they are limited by the absence of a control condition, small sample size, and the study context (single clinical setting).

To date, there are eight published studies evaluating the effectiveness of COS-P for parents. Five had very small samples (ns from 1 to 15). None of these included control or comparison groups and all but one used only self-report questionnaires to measure outcomes. Two were single case studies, the first of which showed post-COS-P improvements in parenting stress, perceptions of self-agency and child functioning, and parenting alliance (19). The second case study showed a reduction in attachment insecurity, anxiety and depression symptoms, and perceptions of child internalizing and externalizing behavior problems following COS-P (20). Two other studies (both *n* = 15) showed post-COS-P improvements in parents' self-reported emotion regulation, attributions about the child's behavior and discipline practices (21), and decreases in caregiver helplessness, feelings of fear, anger, and rejection toward the child, and levels of maternal stress (22). One study with a sample of opiate-dependent caregivers of young children (*n* = 8), reported a post-COS-P reduction in caregiver substance use and in depression, anxiety, and stress symptoms (23).

Three larger COS-P evaluation studies have been published recently. One was a multi-site evaluation of community delivery of COS-P (with no control or comparison group; *n* = 131), which focused primarily on the challenges of program delivery in a low socio-economic area in urban Connecticut, USA (24). Maupin and colleagues reported a reduction in caregiver depressive symptoms following COS-P, with a medium effect size, but no changes in caregiver reports of competency, reflective functioning, and the parent-child relationship. Significant implementation challenges were noted, including limited access to the resources needed to run groups (venue, printing facilities, computer equipment), failure to integrate COS-P into clinical caseloads, and limited clinical supervision.

Risholm Mothander and colleagues (25) reported results of a randomized trial (*n* = 52) examining COS-P plus treatment as usual (TAU), compared with TAU alone, in three Swedish infant mental health clinics. Parents in the COS-P group showed significant increases in balanced caregiving representations (interview measure) and in emotional availability (observational measure) 12 months after baseline. There was no significant change in outcome for the TAU-only group in the same period. However, differences between the two groups were not significant.

The largest COS-P study published to date is a randomized controlled trial (RCT) by Cassidy and colleagues (26). Findings were mixed and somewhat difficult to interpret. Analysis of complete data available for 141 mothers in a sample from the U.S. Head Start program, showed two significant main effects and some interesting moderation effects, all with small-medium effect sizes. Compared with the control group, mothers in the treatment condition reported a reduction in unsupportive responses to child distress and their children showed greater inhibitory control (a component of child executive functioning). There were no significant COS-P effects for child attachment security, as measured by the Strange Situation Procedure (SSP), or for parent-reported child behavior problems; however, for mothers with high attachment avoidance (self-reported), treatment group children scored higher on attachment security and lower on disorganization than control group children post-intervention. Those children whose mothers were low on self-reported attachment avoidance scored lower on attachment security than control group children post-intervention. In addition, treatment group children whose mothers scored low on self-reported attachment anxiety *or* low on depressive symptoms had fewer mother-reported internalizing behavior problems post-intervention than control group children (26). These mixed results should be interpreted with caution, given that the moderation analyses were necessarily exploratory due to study design. However, the indication that COS-P may result in greater attachment security and less disorganization in children of mothers who are high on self-reported avoidance is encouraging and warrants further investigation.

This RCT has clear strengths in its gold standard research design and use of multi-modal measures, including parent report as well as observations of child attachment and executive functioning. However, there are limitations in all COS-P studies to date and, viewed together, the findings are promising, but hardly compelling. This is clearly problematic in a context in which government provision of social service funding is increasingly dependent on funded programs being classified as evidence-based (27). Ongoing debate about what constitutes acceptable evidence (27, 28) notwithstanding, there is a clear need for further research with larger and more diverse samples. Moreover, given the extraordinary dissemination and public investment in COS-P training in Australia, there is an urgent need for research evaluating COS-P as it is delivered in these real-world contexts.

### Real World Research

While the RCT is the expected standard for generating evidence of causation (27, 29, 30), there is a growing awareness that evidence generated under laboratory conditions, while necessary, is not sufficient. RCTs often involve participants and environments so carefully controlled (to maximize internal validity) that they are unrepresentative of the real world, in which comorbidity and contextual complexity are the norm (30–35). The reduction of external validity to improve internal validity is partially offset by conducting RCTs in the field (36). However, the substantial time, financial, and staffing resources required to conduct an RCT (35) are beyond the capacity of many real-world settings. Furthermore, RCTs evaluating group interventions like COS-P are inherently more complex and thus even more resource-intensive than those evaluating individual treatments, due to requirements around group scheduling, minimum numbers, etc. (37). Even randomization itself is under scrutiny in psychological and social field research, with feasibility and suitability often questioned. As McCall and Green (2004, p. 8) contend, “publically funded services are never randomly assigned,” and parent choice and attendance at programs may be a key ingredient determining effectiveness. In light of these issues, there is increasing awareness of the need for evidence-*informed* practice (38), drawing on different levels and types of evidence (27, 30, 35, 39).

### Study Context

The current study developed out of a sustained period of engagement with COS-trained practitioners in Australia. The first step was a pilot survey of practitioners that aimed to investigate the dissemination and implementation of Circle of Security approaches and to identify unmet needs and key issues that required further research and/or evaluation. A link to an anonymous questionnaire was distributed to an email list of professionals who had completed any form of Circle of Security training: 614 respondents began the survey and 521 returned sufficient information for analysis. Of these, 455 (87.3%) had completed the COS-P 4-day training.

Key learnings from these survey responses were that the COS-P intervention was being offered in diverse ways (group/individual) to diverse populations, including families involved with the child protection system and families experiencing socioeconomic disadvantage, child behavioral challenges and/or parent mental health problems, in addition to parents in universal care settings. Responses indicated that COS-P was widely offered by services for women with postnatal depression (PND). Exploring the effectiveness of the intervention for women with PND is a key objective of the current study. The incorporation of COS-P into PND treatment protocols follows empirically-based recommendations that effective interventions for PND should include parenting-specific adjuncts to PND treatment. The well-documented adverse impacts of PND on the child and the parent-child relationship are believed to be predominantly mediated through impaired parenting (40–42) and studies of PND treatments have indicated that, while the mother's mood disorder can be successfully treated, remission of symptoms is not sufficient to improve parenting capacity or outcomes for children (43, 44).

COS practitioner survey responses also indicated that there was little systematic evaluation of COS-P in practice. Where evaluation was undertaken, it was mainly limited to informal observations and follow-up discussions with parents. When validated measures were used, the tools were mostly routine therapy outcome measures, such as mood state measures and the Strengths and Difficulties Questionnaire (SDQ) (45). Responses to open-ended survey questions further indicated that practitioners wanted guidance on: (a) which measures should be used to evaluate program effectiveness; (b) suitability and triage considerations for families with different risk profiles; and (c) compatibility and sequencing of the intervention in relation to other treatments being offered (e.g., treatments explicitly targeting depression). The current study seeks to address some of these issues.

### The Current Study

The primary aim of the current study is to examine the effectiveness of COS-P for caregivers who present to early parenting support services with parenting concerns, often in the context of PND. Study outcomes have been selected with reference to a recently developed theory of change for COS-P (46), which proposes that COS-P works to improve aspects of caregiving that may be necessary prerequisites for secure attachment, including caregiving representations (i.e., how the caregiver thinks and feels about the child, themselves as a caregiver, and their relationship with the child) and child-focused mentalization (the ability to be aware of and make inferences about mental states of self and child, and their impact on behavior). These components of relational caregiving capacity are theorized primary outcomes of COS-P. Changes in parent behavior, and in child attachment and/or behavior are not directly targeted by the intervention, but may be longer-term outcomes of targeted improvements in caregiving, and thus are considered secondary outcomes (46).

We aim to establish if COS-P is effective in building caregiving capacity through an increase in (a) positive representations of the child and self as caregiver, (b) more accurate caregiver mentalization, (c) more responsive caregiving behavior, and (d) reduction of caregiver depression symptoms. We hypothesize that caregivers receiving COS-P will show greater improvements in these areas than caregivers in a waitlist condition.

Given that COS-P research to date includes disparate (and often small) samples with a range of risk factors, we also intend to examine whether socio-demographic (e.g., caregiver language background, gender, education level, child age) and psychosocial (e.g., severity of depression symptoms) risk factors moderate response to the intervention, to extend knowledge of what works for whom. Due to limited empirical data available on COS-P outcomes, we do not posit directional hypotheses regarding the moderating effects of examined demographic and psychosocial risk factors.

In addressing these aims, we will trial a user-friendly evaluation tool assessing primary outcomes in line with the above COS-P theory of change, which may enable scaled measurement of COS-P outcomes through pooling of data from multiple sites. In addition, we will build research capacity within the study sites by training and supporting clinicians in research procedures, including participant recruitment and administration of study measures.

## Methods and Analysis

### Design

This study is a multi-site non-randomized controlled effectiveness study of COS-P, with treatment and waitlist control group participants undergoing assessment at two time points. The multi-site design both reflects the broad dissemination of COS-P and enables recruitment of sufficient participants to meet sample size requirements (see power analysis, below). The study design was determined in consultation with the study sites (see study setting, below); senior managerial staff indicated willingness to support incorporation of the study into their service, but maintained that they could not accommodate a randomized trial. Thus, participant allocation to treatment and waitlist control conditions will not be randomized, but dependent on the scheduled timing of the COS-P group in which they are enrolled. At study entry, participants whose COS-P group will commence within 7 weeks will be allocated to the treatment group. Participants whose COS-P group will commence eight or more weeks hence will be offered a place in the waitlist control group. Circumstances that may contribute to the latter include a long COS-P waiting list at the study site, registering just after a COS-P group has been filled or has started, inability to attend the next available group due to scheduling clashes, being assigned to a group that is subsequently canceled due to insufficient numbers, and the long gap between groups over the summer shutdown period. However, both treatment and control group participants must be determined to be “COS-P-ready” according to standard clinical procedure prior to their participation in the study. Waitlist control group participants will be free to engage with other forms of treatment or support within and outside of the organization prior to commencing the group. This study has been approved by the relevant university, health department and service-specific ethics committees (Macquarie University Human Research Ethics Committee: 5201600788; St John of God Healthcare Human Research Ethics Committee: 1153; Sydney Local Health District Ethics Review Committee: HREC/17/RPAH/285 & SSA/17/RPAH/432; ACT Health Human Research Ethics Committee: ETH.9.17.221E).

### Study Setting

The study will be undertaken in collaboration with four community child and family health organizations (study sites) in two Australian cities located in separate states/territories. There are two study sites in each city. Three of these organizations have an explicit focus on perinatal mood problems, all offer COS-P in their suite of services for families with young children (aged 0-5) and all expressed an interest in participating in a collaborative evaluation study. See Table 1 for site details. All study sites routinely deliver COS-P groups, generally four times per year during school terms. All sites offer COS-P to current clients, and two also make the program available to parents from the community. One site delivers COS-P to clients only toward the end of other treatment, whereas the other three do not specify timing for the intervention. In all cases, group facilitators use their clinical judgement to assess suitability for the group, based on prior casework and/or a pre-group interview (face-to-face or by phone).

**Table 1:** Overview of study sites.

	**Site 1 Tresillian Family Care Centres**	**Site 2 Raphael Services NSW St John of God Healthcare Social Outreach**	**Site 3 ACT Health Perinatal and Infant Mental Health Consultation Service**	**Site 4 Marymead Centre for Early Life Matters**
Type of service	Early parenting support	Perinatal and infant mental health	Perinatal mental health	Early parenting support
Referral pathway/s	•Health professionals •Self-referral for groups	•General practitioners and medical specialists	•Health professionals	•Health professionals •Education professionals •Self-referral
Accessed by parents with…	Parenting challenges, often around feeding, sleeping, settling, adjustment & associated perinatal mental health issues	Mental illness in the perinatal period (pre-conception to index child age 4)	Perinatal mood disorders (pregnancy to 12 months post-partum)	Concerns about parenting, adjustment, mental health, or child relationship, emotional, or behavioral issues
Child age range	0–5 years	Pre-conception to 4 years old	0–5 years	0–8 years
Professional staff	•Nurses •Social Workers •Psychologists •Psychiatrists/Registrars •Pediatricians •GPs	•Psychiatrists/registrars •Clinical Psychologists •Social Worker •Mental Health Nurses	•Medical Officer •Psychiatrists/Registrars •Psychologists •Social Workers •Occupational Therapists •Nurses	•Psychologists •Social Workers •Counselors
Where does COS-P fit into treatment?	•Referral pathways from residential & day stay services •Stand-alone parenting program	•Offered toward end of treatment	•During and toward end of treatment	•Stand-alone parenting program
Who delivers COS-P?	•Allied Health staff •Nurses •Psychiatry Registrars (rarely)	•Psychiatrist/registrar •Social workers •Mental health nurses	•Allied Health staff •Mental health nurses	•Psychologists •Social workers •Counselors
Who can access COS-P?	•Clients •Parents in the community	Clients only	Current and recent clients only	•Clients •Parents in the community
Cost of COS-P	AUD88 (waived in cases of financial hardship)	No cost	No cost	No cost

Following development of a research proposal, meetings were held with management (and lead clinical staff, in some cases) at each organization, to discuss the study and its feasibility in each setting. The study design, procedures, and measures were finalized in collaboration with representatives of each of the study sites.

### Participants

Eligible participants will be primary caregivers and/or their partners, with a child aged 0–60 months (at study entry), who are registered to attend a COS-P group at one of the study sites during the 18–24 month study period. Study exclusion criteria (an acute disorder or one likely to limit participation; insufficient English proficiency to complete study measures) are, in fact, also site exclusion criteria for referral to COS-P groups. They are routinely assessed at the time of engagement with the organization and also during routine pre-group-enrolment screening. Any participant whose assessment indicates risk to parent or infant will be triaged into other appropriate treatments. Thus, the single study-specific exclusion criterion is having attended COS-P sessions prior to study enrolment. Participants will receive no reimbursement for study participation.

### Procedure

All eligible clients will be offered the opportunity to participate in the study as soon as is practical after their registration for COS-P. In most cases, administrative or clinical staff will explain the study and invite participation during their routine pre-group contact with clients. In both cities, a locally-based member of the research team will provide study oversight and research support, including assistance with participant recruitment and administration of study measures, as required by study sites.

Study measures will be administered by site clinicians and members of the research team, all of whom will receive related training and written instructions. Personnel administering measures in each case will depend on site capacity. Two study questionnaires will be administered to all study participants; interviews and observational procedures will be administered only to the subsample of participants who consent to and can complete these additional measures within the required timeframe. Treatment group participants will complete study measures a maximum of 2 weeks before the first session (Time 1) and a maximum of 2 weeks after the final session (Time 2) of their COS-P group. Those completing only study questionnaires will complete them at the relevant COS-P session (i.e., Time 1 at the start of session 1 and Time 2 at the end of session 8). Waitlist control group participants will complete both Time 1 and Time 2 study measures within the same 7 to 11-week timeframe, before they commence COS-P. Waitlist-control group participants completing only questionnaires will complete them onsite, if possible, otherwise they will be mailed hard copies or emailed individualized links to online versions of the Time 1 and Time 2 questionnaires. The latter process will be managed by the first author, using the university's password-protected Qualtrics platform. A separate record of individualized links by Client ID will enable matching of Time 1 and Time 2 data, and linking with clinical file data. De-identified questionnaire data for these participants will be stored securely in Qualtrics. All participants completing additional interview and/or observational procedures will complete these assessments at their study site or in their home, depending on site capacity, and participant convenience. For participants completing the observational assessment, time of day will be kept consistent between Time 1 and Time 2 assessments, to the extent possible considering parents' availability constraints and the unpredictability of infant/child sleep-wake cycles. See Figure 2 for study flow.

**Figure 2:** Flowchart detailing participant flow through study, including timing of measures and intervention.

The study interview will be audio recorded and will take approximately 1 h to complete. Time 1 and Time 2 interviews for each participant will be administered by two different members of the research team, as required by the nature of the interview and associated coding system. Since the time between interviews is relatively short, and participant elaboration vs. more truncated responses can be meaningful in coding, it is important that participants do not reduce the detail in their Time 2 answers due to a perception of interviewer familiarity from Time 1. While we acknowledge the potential for interviewer-related bias with this approach, evaluation of test-retest reliability of a similar narrative interview with different interviewers at each time point found no interviewer effects (47, 48). To maximize consistency of administration, and thus minimize the risk of systematic bias in the current study, interviewers will undergo training and receive regular research support (see below), will use a standardized interview template and written protocol, and will undertake a mix of Time 1 and Time 2 interviews for both treatment and control group participants. For treatment group participants, where possible, the site clinician scheduled to facilitate their COS-P group will administer Time 1 (pre-group) interviews and video assessments, and a member of the research team will administer Time 2 (post-group) interviews and video assessments. For control group participants, administration personnel will be reversed. A participant's COS-P group facilitator will never administer their post-group study interview, to reduce risk of associated response bias.

The observational procedure is a 5-min caregiver-child free play interaction (video recorded), detailed in a written protocol with illustrations. Caregivers will be given the instruction, *play with your child as you would if you had a spare 5- minutes at home*. Two consistent toys will be provided—a baby doll with clothes, and a train with detachable carriages—and caregivers will be told they may use these toys if they wish. For children up the age of 12 months, caregivers will be requested to place the child in a fixed seat (e.g., car chair or high-chair) and to sit opposite the child with their face at the child's face level. For children aged 13 months and up, caregivers will be requested to sit opposite their child on the floor.

Pre-specified additional participant data will be retrieved from clinical files at each site by senior clinicians/managers and sent to the research team using client study ID only (permission granted as part of study consent process). These data comprise country of birth, living situation (single, cohabiting), number of children, history of mental health problems (if disclosed), current medication for mental health disorder, and (via chart audit) additional treatment/service received during study participation, including non-group COS-P content. Study processes will be documented to enable a *post-hoc* process evaluation (37).

#### Training of Researchers and Clinicians at Study Sites

To enable reliable administration of study measures, and to maximize study participation and promote a research culture in study sites, researchers and participating site clinicians will be provided with training in and support for participant recruitment, and administration and clinical application of all study measures. This will include 1-day training in administration of the study narrative interview, incorporating an introductory explanation of the coding system and discussing clinical implications of different types of responses, facilitated by an expert in the interview who developed the coding system (third author). Regular face-to-face site meetings and/or videoconferencing will be held to monitor the study procedures and recruitment progress, and to address implementation challenges. All participating clinicians must be trained and certified to deliver the COS-P intervention prior to their participation in this study.

### Intervention

At all study sites, COS-P will be facilitated to groups of parents according to the original program manual (6) utilizing the associated DVD, over 8 weekly 90 to 120-min sessions; one manual chapter (with associated DVD content) to be completed *per session*. Following standard COS-P research practice, intervention completion will be defined as attendance at a minimum of six sessions (Neil W. Boris MD, Research Liaison and Medical Director—Circle of Security International, personal communication, 15 August 2017).

To maximize intervention fidelity, collaborating study sites have been chosen, in part, for their adherence to the COS-P manual in their routine delivery of COS-P. Beyond this, as the study aims to evaluate COS-P-as-delivered, intervention fidelity will be assessed by the research team, through post-group interviews with each COS-P facilitator (see interview details below).

### Measures

Study measures were selected for minimum participant burden to ensure feasibility for high-volume outpatient community health settings, and based on their suitability across a broad child age range, their alignment with aspects of parenting targeted by the intervention, and existing evidence of validity, reliability and utility for both research and clinical work.

#### Primary Outcomes

Primary outcomes are caregiving representations, assessed through a self-report questionnaire and a narrative interview, and caregivers' parental mentalization, assessed through a self-report questionnaire, and from caregiver language during a narrative interview and observed caregiver-child interaction.

##### Composite caregiving questionnaire

The CCQ was developed to evaluate primary COS-P outcomes; specifically, components of caregivers' self-reported caregiving representations and parental mentalization. With a view to keeping the questionnaire brief and minimizing repetition, subscales from several validated questionnaires were combined, with their authors' permission. The original rating scales were retained for each subscale. In prior research using the original measures, subscale totals have commonly been reported in addition to (and sometimes, instead of) overall totals. Following initial development, three study sites (sites 1, 2, and 3) piloted the CCQ with COS-P group participants. Feedback from participants, clinicians and service managers led to wording refinements including replacement of “mother” or “parent” with “caregiver,” and providing simpler explanations for some words and phrases that may be unfamiliar to non-native-English speakers. The final study version of the CCQ has 43 items, incorporating:

- 12 items from two subscales of the tool to Measure Parenting Self-Efficacy (TOPSE)^1^ (49), scored on a 10-point scale, exploring:
  – empathy and understanding (six items; e.g., *I understand my child's needs*), and
  – emotion and affection (six items; e.g., *I am able to show affection to my child*)
- six items from the parenting questionnaire used in the Longitudinal Study of Australian Children (LSAC) (50), exploring:
  – hostile parenting (five items; e.g., *When this child cries, he/she gets on my nerves*) scored on a 10-point scale
  – parent overall rating of child difficultness (from the Australian Temperament Project (51)); single item; *Compared to the average child, do you think your child is…*) scored on a 5-point scale, ranging from *Much less difficult* to *Much more difficult*
- seven items from the Caregiving Helplessness Questionnaire (Mother Helpless subscale, CHQ (52)); e.g., *When I am with my child, I often feel out of control*) scored on a 5-point scale
- the full 18-item Diamond Maternal Reflective Functioning Scale [DMRFS; (53); e.g., *I think about what my child may be thinking or feeling*] scored on a 4-point scale

Preliminary reliability and validity assessments for the subscales, as combined in the CCQ, were undertaken on a pilot sample of 81 parents. Internal consistency was very good; Chronbach's alpha coefficients ranged from 0.78 (TOPSE emotion and affection) to 0.88 (TOPSE empathy and understanding, and LSAC hostility). Associations among subscales (plus depression symptoms) aligned with theoretical expectations, but they were moderate, confirming that the different subscales captured different aspects of parenting: e.g., hostility was positively correlated with caregiving helplessness (0.68) and depression symptoms (0.54) and negatively correlated with empathy and understanding (−0.34); caregiving helplessness was negatively correlated with empathy and understanding (−0.57); and positively correlated with depression symptoms (0.57). Self-reported caregiving representations and parental mentalization will be compared with assessments of these outcomes using validated interview and observational measures during this study, as part of the ongoing CCQ validation process.

##### The circle of security interview

Augmenting the CCQ, the Circle of Security Interview [COSI; (9)] will enable a more in-depth assessment of caregiving representations. The COSI is based on two widely validated instruments to assess attachment and caregiving representations, respectively, the Adult Attachment Interview (AAI) (54); and the Parent Development Interview (PDI) (55). The COSI forms part of the 20-week COS-I treatment protocol, and differs from the two source measures by including direct questions to the parent about their experience of the Strange Situation Procedure (SSP). The final question asks the caregiver what they hope the target child learns from being parented by them. Like the AAI and the PDI, the COSI is a narrative interview, designed to “surprise the unconscious” [(54), p. 19], and is thus less prone to response bias than a questionnaire.

In the current study, the questions related to the SSP will be omitted. Interviews will be audio recorded and transcribed, and de-identified transcripts will be used for coding. Responses to the questions exploring perceptions of self in the caregiving role and relationship with the target child will be coded using a coding system developed by Huber and colleagues (16). This eight-scale system comprises two affect dimensions, reflecting the caregiver's feelings about the child and/or their relationship, and six dimensions reflecting the caregiver's self-perception in the caregiving role (16). The system shows promising validity, with theoretically expected associations between one subscale (“weak”) and observed dimensions of attachment (negatively correlated with attachment security and positively with attachment disorganization) (16) and between the total representations score and parental mentalizing (positive correlation with appropriate mind-related comments) (56).

##### Interview and observational assessments of caregiver mind-mindedness

To supplement the CCQ, more in-depth measures of parental mentalization will be included. The mind-mindedness interview question (*Please describe your child*) (57) will be added to the COSI. Parent spontaneous descriptions of their child, together with parent language during the 5-min videotaped caregiver-child interaction, will be transcribed and coded, respectively, for representational and observational mind-mindedness (58, 59), according to Meins and Fernyhough's coding manual (57). Mind-mindedness is a measure of parental mentalization specific to the child (60), and one of the most feasible and cost-effective to administer and code (61). Mind-mindedness has shown consistent associations with parental sensitivity and child attachment (61).

#### Secondary Outcomes

The two secondary study outcomes are caregiver-child interaction quality, assessed from observed caregiver-child interaction, and caregiver depression symptoms (also being tested as a moderator), assessed through a self-report questionnaire.

##### Caregiver-child interaction coding scheme

Caregiver-child interaction videos will be coded using an adaptation of the coding scheme for assessing maternal interactive style developed by Calkins and colleagues (62) and validated for short interactions by Bernier and colleagues (63). The two original versions of the scheme (one for mothers of 5- and 10-month-old infants, and one for mothers of 24-, 36-, and 48-month-old children) were combined to form a single coding scheme suitable for use with children from infancy to 5 years of age, including guidance on developmental variations. The adapted coding scheme comprises four scales for rating caregiver behavior and one scale for rating child behavior. Three of the caregiver scales were part of in the original measures—sensitivity (previously called Facilitates Attention), Intrusiveness, and Hostility (previously called Negative Affect). An additional caregiver scale, Autonomy Support, based on work by Whipple and colleagues (64), and one child scale, Child Inclusion of Caregiver, have been added. Following the approach used by Calkins and colleagues (62) each 5-min video will be coded in ten 30-s intervals. Ratings for each scale will be summed across the 10 intervals and then divided by 10 to give a mean value. Following initial adaptation, the new coding scheme will be refined during group coding of the first 10 video cases by the three study coders.

##### Edinburgh postnatal depression scale (EPDS)

The EPDS (65), already in routine use at three of the four study sites, will be used to assess depression symptoms before and after the group. This well-validated measure comprises 10 questions exploring possible symptoms of depression, designed to be suitable for use in the postnatal period as few items refer to maternal sleep and appetite disturbances which are to be expected with a newborn. Although the EPDS was developed to screen for depression in antenatal and postnatal women, it has been validated for the assessment of mothers of preschool-aged children (66), fathers (67), and adults in the general population (68). While depression symptoms are not an explicit primary or secondary target of COS-P, there is some evidence from the limited COS-P research to date that depression symptoms are improved following COS-P (24, 69), and maternal depression is commonly examined as a moderator of the effectiveness of attachment-based interventions (26).

#### Monitoring Intervention Fidelity

##### COS-P fidelity interview

A brief structured interview was developed to track program fidelity during this study. Questions administered to all COS-P facilitators at the end of each group will probe adherence to the COS-P manual and DVD clips. Any content excluded or added will be noted. This interview will also provide an opportunity for facilitators to share any factors they noted during the group that might influence intervention completion or outcomes for specific participants, e.g., divorce, separation, or death of a significant other during the course of the group, presence of a partner in the group, etc.

#### Ensuring Caregiver and Child Safety

As all study participants will be clients of a clinical service, they will be allocated to a case manager or clinician at that service, and their mental health and well-being will be routinely monitored. Potential study participants will be excluded from the group (and therefore, the study) by clinical staff if they are too impaired due to severe mental illness, suicidality, or psychosis, and referred for more intensive support. Given different service types and resource levels, some services provide this internally, while others will refer externally. In addition to routine monitoring, Time 1 and Time 2 EPDS assessments will be used to detect mental health symptom severity and risk. Study sites have established protocols and pathways for parents that score in the likely-to-be-depressed range (>12) or endorse item 10 (risk item). In addition, during COS-P group participation, clinicians routinely assess and monitor for mental health symptoms, risk to children, and domestic violence, with site-specific protocols in place. In addition to established site protocols for ensuring caregiver and child safety, there will be regular communication between the research team and clinical and managerial staff at the study sites. At clinical service discretion, parents with significant risk or safety issues, and/or who require more intensive, individual interventions, will be withdrawn from the study and referred as above.

### Sample Size Calculation

Power analyses were conducted using G^*^Power 3.1 (70). Based on preliminary CCQ data for the first 67 intervention group participants, a total sample size of 128 was indicated to detect a medium intervention effect with 80% power and an error level of 0.005 (for multiple comparisons). Assuming an attrition rate of 20%, we aim to recruit a total of 154 participants to complete study questionnaires. Sample size for the interview and observational study measures was calculated based on analysis of data from the COSI interview in a previous comparable study (16). While there was a large intervention effect on caregiving representations in that study, it is estimated the effect size will be smaller in the current study given the shorter duration and lower intensity of the intervention. To detect a medium effect size with 95% power and an error level of 0.05, assuming a Time 1–Time 2 correlation of 0.5, a sample size of 40 was indicated. Assuming an attrition rate of 20%, we aim to include a subsample of 48 participants completing interview and observational study measures (COSI and/or videotaped caregiver-child interaction) in addition to questionnaires.

### Data Analysis

Given that this is not a randomized trial, an intention to treat analysis is not essential. To maximize understanding of what works for whom, we seek to measure the intervention effect on those participants who actually receive the intervention—and we also seek to understand the factors that influence completion and non-completion of COS-P, as well as variations in response (71). Thus, data in this study will primarily be analyzed to measure the treatment effect on participants who received COS-P as intended. Complete Time 1 and Time 2 data for study participants who attend at least six of the eight COS-P sessions will be included in these analyses, together with data from clinical files and information collected during facilitator fidelity interviews, if appropriate. For participants who (a) attend 5 or fewer COS-P sessions and/or (b) do not complete Time 2 measures, treatment effect will not be measured; only Time 1 data, clinical file data and information collected during facilitator fidelity interviews will be analyzed, to explore whether characteristics of these caregivers distinguish them from completers and/or influence failure to complete the intervention.

Analyses will be conducted using SPSS Version 26 (72). Descriptive analyses will be used to profile and compare the characteristics of the treatment and waitlist control groups in the four participating sites. Bivariate correlations and independent samples *t-*tests will be used to explore relationships among the outcome variables and any potential covariates. As group allocation is not randomized, and recruitment is undertaken across four sites with different characteristics, the two groups may differ on distribution of demographic and risk factors which may impact on intervention effects. Baseline comparability will be assessed using independent samples *t*-tests (for continuous variables) and chi-square tests of independence (for categorical variables). Mixed design ANOVA will be used to control for any observed differences in baseline characteristics. Due to anticipated differences among participant cohorts from the four different sites, child age and depression symptoms (EPDS score at Time 1) will be included as *a priori* covariates. If sample size and composition allow, results will be stratified by site.

## Discussion

Widely disseminated yet strikingly under-researched, COS-P is a program with evident appeal and potential, but little evidence of effectiveness. This study is designed to help address this evidence gap. It is the first COS-P effectiveness study in Australia, one of the first worldwide, and one of the few to utilize a control condition. The collaboration of four clinical services currently offering COS-P to clients provides a valuable opportunity to measure program effectiveness in these real-world settings.

Given the complexity of the study context, several challenges are expected, which will need to be managed at different stages of the study. Firstly, there is increased potential for baseline differences among treatment and control group participants due to the non-randomized design. Although it cannot match the rigor of an RCT, the repeated measures design enables investigation of potential differences between groups in preliminary analyses, so the influence of any known differences can be controlled in main analyses, reducing potential confounds. However, we acknowledge the possibility of unknown confounding variables. Secondly, the differences between study sites with respect to client numbers, characteristics, referral pathways, treatment protocols (outside of COS-P), and child age, may increase sample heterogeneity and may affect generalization of findings. If sample size allows, results will be stratified by site, but we acknowledge that this may not be possible. In addition, staff turnover, clinical loads, and/or lack of clinician buy-in to the study may reduce research capacity in some sites at some stages of the study. Inherent site differences and staffing challenges may lead to unequal participant numbers across the four sites, complicating data analysis. Finally, we acknowledge it is possible that elements of the Circle of Security model are diffused throughout the study sites, informing broader practice, which may compromise a clear distinction between the COS-P treatment and any TAU provided to the waitlist control group. These challenges will be carefully documented and considered in study analyses and interpretation and discussion of results.

Despite the expected challenges, it is anticipated that this study will contribute valuable evidence on the effectiveness of COS-P. While the non-RCT design will not deliver the strength of evidence required to comprehensively address the COS-P evidence gap, it will provide information on the impact of COS-P, as delivered within specialized parenting and perinatal mental health services in Australia for caregivers experiencing parenting challenges in the early parenting period. The comparatively large sample, controlled design, and use of rigorous outcome measures, will ensure that study findings can strengthen the COS-P evidence base. If findings are inconclusive, the process evaluation will provide an opportunity to advance understanding about intervention provision and research in complex real-world settings, and inform the design of future studies. In addition, the use of a measure that has been used previously in a study of COS-I (16) will enable a comparison of the effectiveness of both COS interventions. This evidence will add to our growing understanding of what works for whom in perinatal mental health and broader parenting and early childhood service provision.

## Dissemination and Data Sharing

The de-identified results of the research across the four services, will be made available to participating services through webinars, videoconferencing and/or face-to-face meetings. In addition, a face-to-face visit (or videoconference) will be provided to each service to present and discuss their own results. This study will generate evidence about the effectiveness of Circle of Security Parenting program, including for parents who are experiencing postnatal depression. Dissemination of findings to other parenting services, perinatal mental health services and state and federal policy makers will occur through our well-established networks of knowledge exchange and partnership. Dissemination of findings will also occur through academic publication [following STROBE reporting guidelines; (73)], and national and international conferences.

## Ethics Statement

The studies involving human participants were reviewed and approved by the relevant university, health department and service-specific ethics committees (Macquarie University Human Research Ethics Committee: 5201600788; St John of God Healthcare Human Research Ethics Committee: 1153; Sydney Local Health District Ethics Review Committee: HREC/17/RPAH/285 and SSA/17/RPAH/432; ACT Health Human Research Ethics Committee: ETH.9.17.221E). The patients/participants provided their written informed consent to participate in this study.

## Author Contributions

A-MM, CM, AH, RR, and EH were responsible for conception and design of the original study, and have contributed to ongoing study design and development. A-MM is managing rollout of the study, in consultation with CM. RR is providing study oversight in Canberra. A-MM wrote the first and successive drafts of this manuscript. All authors were involved in critically revising the manuscript and have read and approved the final manuscript. All authors contributed to the article and approved the submitted version.

## Conflict of Interest

A-MM facilitates COS-P parent groups as part of her work with a non-profit organization. AH facilitates COS-P facilitator training once annually, for which she receives payment from Circle of Security International. The remaining authors declare that the research was conducted in the absence of any commercial or financial relationships that could be construed as a potential conflict of interest.

## Footnotes

^1^University of Kent. Available online at: http://topse.org.uk (accessed February 29, 2016).
